# MicroRNA-203 inhibits malignant melanoma cell migration by targeting versican

This article has been retracted.

**DOI:** 10.3892/etm.2014.1708

**Published:** 2014-05-12

**Authors:** PINGYUAN BU, PING YANG

**Affiliations:** Department of Burns, The Third Xiangya Hospital of Central South University, Changsha, Hunan 410013, P.R. China

**Keywords:** malignant melanoma, microRNA-203, versican, migration

## Abstract

MicroRNA (miR)-203 has been demonstrated to function as a suppressor in tumorigenesis. Recently, miR-203 was reported to play a role in malignant melanoma (MM); however, the detailed function of miR-203 in MM remains unclear. In the present study, the expression of miR-203 was shown to be significantly downregulated in MM tissues when compared with normal adjacent tissues. Based on a bioinformatic prediction, versican was further identified as a novel target of miR-203, and the expression of versican was markedly increased in MM tissues. Inhibition of miR-203 increased the protein expression of versican, while upregulation of miR-203 inhibited the protein expression of versican in MM A375 cells. In addition, the upregulation of versican significantly promoted A375 cell migration; however, upregulation of miR-203 suppressed A375 cell migration. The present study further investigated whether miR-203 was involved in versican-mediated A375 cell migration, and the results indicated that upregulation of miR-203 significantly inhibited A375 cell migration, which was impaired by overexpression of versican. These observations indicated that versican functions as a downstream effector in miR-203-mediated MM cell migration. Therefore, the results demonstrated that miR-203 exhibited an inhibitory effect on MM cell migration via directly targeting versican, thus, may become an effective inhibitor for MM metastasis.

## Introduction

Malignant melanoma (MM) is a very aggressive skin cancer that has been shown to be a continuing health threat. MM is the fifth most common cancer in males and the seventh most common malignancy in females (1). A previous study estimated that the incidence of MM has increased by 3.1% in one year (2). In addition, the incidence of MM is increasing in males and females more than any other malignancy, with the exception of lung cancer (1). Therefore, developing effective targets and agents for the treatment of MM is urgently required.

MicroRNAs (miRNAs) are a family of endogenous, small (18–25 nucleotides in length), noncoding, functional RNA molecules, which can induce post-transcriptional silencing by directly binding to a target sequence in the 3′-untranslated region (UTR) of their target RNAs (3). Recently, a number of miRNAs have been demonstrated to play key roles in melanoma (4,5). A recent study applied an Illumina next-generation sequencing platform to conduct an in-depth analysis of the miRNA transcriptome in MM with matched normal skin, and demonstrated that miR-203, -204-5p, -205-5p, -211-5p, -23b-3p, -26a-5p and -26b-5p were significantly decreased in MM (6). Among these miRNAs, miR-203 has been shown to play a suppressive role in multiple types of human malignancies. For example, Yu *et al* showed that miR-203 suppressed the proliferation and self-renewal of esophageal cancer stem-like cells by targeting BMI1 (7). In addition, Wang *et al* reported that miR-203 downregulated the proliferation and migration of lung cancer cells by inhibiting protein kinase C-α (8). Recently, miR-203 was hypothesized to play a pivotal role in MM via reducing melanosome transport and promoting melanogenesis by targeting KIF5B (9). An additional study revealed that the loss of miR-203 expression at the invasive front of primary cutaneous melanoma was associated with increased tumor thickness and disease progression, indicating that miR-203 may play a crucial role in the regulation of MM cell invasion (10).

Versican is a hyaluronan-binding, extracellular chondroitin sulfate proteoglycan located within the extracellular matrix (ECM). Due to its ability to interact with cell surface components and the ECM, versican was found to play a crucial role in tumor cell attachment to the interstitial stromal matrix of tumors. Previously, versican was shown to be directly targeted by miR-143, and the repression of versican by miR-143 was involved in platelet-derived growth factor BB-induced migration of smooth muscle cells (11). Accordingly, we hypothesized that the role of versican in MM cell migration may also be associated with miRNAs. However, to the best of our knowledge, the association between versican and miRNAs in MM has not been previously reported. In the present study, we aimed to investigate the detailed role of miR-203 and versican in the regulation of MM cell migration.

## Materials and methods

### Tissue specimen collection

All experimental protocols were approved by the Ethical Committee of the Third Xiangya Hospital of Central South University (Changsha, China). In total, 24 melanoma tissues, as well as matched adjacent normal tissues, were obtained from patients at the Department of General Surgery, the Third Xiangya Hospital of Central South University. Informed consent was provided by the patients involved in the study. Following surgical removal, tissue samples were immediately frozen in liquid nitrogen.

### Cell culture

Human malignant melanoma A375 and human normal skin HaCaT cell lines were obtained from the Cell Bank of Central South University. Cells were cultured in Dulbecco’s modified Eagle’s medium (DMEM; Invitrogen Life Technologies, Carlsbad, CA, USA) supplemented with 10% fetal bovine serum (FBS; Invitrogen Life Technologies) at 37°C in a humidified incubator containing 5% CO_2_.

### Quantitative polymerase chain reaction (qPCR)

Total RNA was extracted with TRIzol reagent (Invitrogen Life Technologies), in accordance with the manufacturer’s instructions. For the analysis of mRNA expression, a *Taq*Man Reverse Transcription kit (Thermo Fisher Scientific, Waltham, MA, USA) was used to convert RNA into cDNA, following which qPCR was performed using a Power SYBR Green kit (Thermo Fisher Scientific) with an ABI 7500 thermocycler (Invitrogen Life Technologies). Glyceraldehyde-3-phosphate dehydrogenase (GAPDH) was used as an endogenous control. The primers used were as follows: Versican forward, 5′-GTAACCCATGCGCTACATAAAGT-3′ and reverse, 5′-GGCAAAGTAGGCATCGTTGAAA-3′; GAPDH forward, 5′-ACAACTTTGGTATCGTGGAAGG-3′ and reverse, 5′-GCCATCACGCCACAGTTTC-3′. For the analysis of miRNA expression, an ABI miRNA reverse transcription kit (Applied Biosystems; Thermo Fisher Scientific) was used to convert RNA into cDNA, according to the manufacturer’s instructions. Next, qPCR was performed using an miRNA qPCR Detection kit (GeneCopoeia, Rockville, MD, USA) with an ABI 7500 thermocycler. The U6 gene was used as an endogenous control. For mRNA and miRNA, relative expression levels were analyzed using the 2^−ΔΔCt^ method.

### Western blot analysis

Tissues or cells were solubilized in cold radioimmunoprecipitation lysis buffer. Proteins were separated with 12% SDS-PAGE and transferred onto a polyvinylidene difluoride membrane, which was then incubated with Tris-buffered saline Tween-20 containing 5% skimmed milk at 4°C overnight. Next, the membrane was incubated with rabbit anti-versican and mouse anti-GAPDH primary antibodies (Abcam, Cambridge, UK) at room temperature for 3 h. Following washing with phosphate-buffered saline Tween-20 (PBST) three times, the membrane was incubated with goat anti-mouse or goat anti-rabbit secondary antibodies (Abcam), respectively, at room temperature for 1 h. The membrane was washed again with PBST three times. An enhanced chemiluminescence kit (Pierce Biotechnology, Inc., Rockford, IL, USA) was used for chemiluminescent detection. Relative protein expression was analyzed with Image-Pro Plus software 6.0 (Media Cybernetics, Inc., Rockville, MD, USA), and was represented as the density ratio against GAPDH.

### Transfection

Transfection was performed using Lipofectamine 2000 (Invitrogen Life Technologies), according to the manufacturer’s instructions. For miR-203 functional analysis, melanoma A375 cells were transfected with scrambled miRNA as a negative control, miR-203 mimics or miR-203 inhibitor (Invitrogen Life Technologies). For versican functional analysis, human melanoma A375 cells were transfected with a pcDNA3.1-versican plasmid.

### Dual luciferase reporter assay

A mutant type 3′-UTR of versican was generated using a Quick-Change Site-Directed Mutagenesis kit (Stratagene, Inc., La Jolla, CA, USA). The wild type and mutant type 3′-UTRs of versican were inserted into the psiCHECK™2 vector (Promega Corportation, Madison, WI, USA). Next, human melanoma A375 cells were cultured to ~60% confluence in a 24-well plate and Cellfectin II reagent (Invitrogen Life Technologies) was used to transfect the A375 cells with the psiCHECK™2-versican-3′-UTR or psiCHECK™2-mutant versican-3′-UTR vectors, with or without 100 nM miR-203 mimics. At 48 h after transfection, the dual luciferase activity levels in each group were examined with an LD400 luminometer (Beckman Coulter, Fullerton, CA, USA). Renilla luciferase activity was normalized against firefly luciferase activity.

### Cell migration assay

For the cell migration assay, 24-well Transwell chambers (Chemicon International, Inc., CA, USA) were used. In each group, a cell suspension (5×10^5^ cells/ml) was prepared in serum free DMEM, and 500 μl DMEM with 10% FBS was added to the lower chamber, while 300 μl cell suspension was added to the upper chamber. Following incubation at 37°C with 5% CO_2_ for 24 h, the non-invading cells were removed and the cells that had passed through the membrane were stained for 20 min, rinsed with water and dried. Five fields were randomly selected under the microscope (Nikon, Tokyo, Japan), and the stained cell number was counted.

### Statistical analysis

Results are expressed as the mean ± standard deviation of three independent experiments. SPSS 18 software (SPSS, Inc., Chicago, IL, USA) was used to perform statistical analysis. Statistical analysis of the differences was conducted using one-way analysis of variance, where P<0.05 was considered to indicate a statistically significant difference.

## Results

### Expression of miR-203 is downregulated in MM tissues

Expression levels of miR-203 were determined in MM and matched adjacent tissues using qPCR. The results showed that the expression of miR-203 in MM tissues was significantly downregulated when compared with the matched adjacent tissues (Fig. 1A). Expression levels of miR-203 were further investigated in normal skin HaCaT cells and MM A375 cells, and miR-203 was found to be significantly downregulated in A375 cells as compared with the HaCaT cells (Fig. 1B). These observations indicate that miR-203 may play a suppressive role in the development and progression of MM.

### miR-203 directly targets the 3′-UTR of versican

Based on a bioinformatic prediction using the software Targetscan (http://www.targetscan.org/), the putative binding site for miR-203 at the 3′-UTR of versican was found to be highly conserved (Fig. 2A). To verify whether versican is a direct target of miR-203, wild type and mutant type 3′-UTRs of versican were generated. A dual luciferase reporter assay was then performed and the results demonstrated that the renilla/firefly value of luciferase activity was significantly reduced in the MM A375 cells cotransfected with the wild type 3′-UTR of versican and miR-203 (Fig. 2B). However, the renilla/firelfy value of luciferase activity in the MM A375 cells cotransfected with the mutant type 3′-UTR of versican and miR-203 exhibited no difference when compared with the control group (Fig. 2B). The observations indicate that versican is a direct target of miR-203 in MM A375 cells.

### Expression levels of versican are increased in MM tissues and MM A375 cells

The mRNA and protein expression levels of versican in MM and matched adjacent normal tissues were further determined using qPCR and western blot analysis, respectively. As shown in Fig. 3A, the mRNA expression level of versican in MM tissues was significantly increased when compared with the matched adjacent tissues. Western blot analysis data further confirmed that the protein expression of versican was upregulated in MM A375 cells when compared with the normal tissues (Fig. 3B). Therefore, versican may play a suppressive role in MM.

### Expression of versican is negatively regulated by miR-203 at a post-transcriptional level in MM A375 cells

To further determine the effects of miR-203 on versican expression in MM cells, MM A375 cells were transfected with miR-203 mimics, miR-203 inhibitor or scramble miRNA. Following transfection, miR-203 expression levels were analyzed in A375 cells. The results revealed that miR-203 expression was upregulated following transfection with miR-203 mimics and downregulated with the inhibitor (Fig. 4A). The protein expression levels of versican were investigated with western blot analysis. As shown in Fig. 4B, the protein expression levels of versican were significantly reduced in MM A375 cells transfected with miR-203 mimics, but upregulated in A375 cells transfected with the miR-203 inhibitor. These observations indicate that miR-203 negatively modulates versican expression at a post-transcriptional level in MM cells.

### Versican has a promoting effect on MM cell migration

Since versican was shown to play a role in the regulation of cell migration (12), the effect of versican on MM A375 cell migration was further investigated. Following transfection of MM A375 cells with the versican plasmid and versican siRNA, the protein expression of versican was analyzed. The results demonstrated that the transfection efficiency was satisfactory (Fig. 5A). It was further demonstrated that overexpression of versican significantly promoted MM A375 cell migration, while siRNA-mediated versican inhibition markedly suppressed A375 cell migration (Fig. 5B). These observations indicate that versican plays a promoting role in MM cell migration.

### Versican functions as a downstream effector in miR-203-mediated inhibition of MM cell migration

As miR-203 was shown to negatively regulate the protein expression of versican by directly targeting the mRNA 3′-UTR, it was hypothesized that miR-203 may play a suppressive role in MM cell migration via the inhibition of versican. Therefore, A375 cells were transfected with miR-203 mimics, or were cotransfected with miR-203 mimics and the versican plasmid. A cell migration assay was then performed and it was found that upregulation of miR-203 significantly inhibited A375 cell migration, which was impaired by overexpression of versican (Fig. 6). These observations indicate that miR-203 inhibits MM cell migration, partially at least, via the downregulation of versican.

## Discussion

It is well established that miRNAs function as key mediators in various biological processes, mainly attributed to their capacity to modulate the expression of target genes at a post-transcriptional level (13,14). Furthermore, deregulation of miRNAs plays a central role in the development and progression of human malignancies. In the current study, the expression level of miR-203 was shown to be significantly decreased in MM tissues when compared with adjacent normal tissues. These observations are consistent with a number of previous studies. For example, Xu *et al* performed miRNA-microarray analysis on MM samples from various stages to identify differentially expressed miRNAs, and showed that miR-203 was differentially expressed between primary and metastatic melanomas (15), indicating that miR-203 may be involved in the progression of MM. Noguchi *et al* examined the expression profile of miRNAs in canine oral MM tissues using a microarray assay and demonstrated that a decreased expression of miR-203 was significantly associated with a shorter survival time (16). In addition, the authors found that the expression of miR-203 was significantly reduced in canine and human MM cell lines (16), consistent with the observations of the present study that miR-203 is downregulated in MM A375 cells as compared with normal skin HaCaT cells. A previous study (10)reported that downregulation of miRNA-203 at the invasive front of primary MM was associated with increased tumor thickness and disease progression. Furthermore, Kozubek *et al* applied an Illumina next-generation sequencing platform to perform an in-depth analysis of the miRNA transcriptome in biopsies of nevi, thick primary and metastatic MM with matched normal skin, and found that miR-203 was among the miRNAs that were markedly downregulated when compared with the control nevi (6). Based on these previous observations and the current results, we hypothesize that miR-203 plays a crucial role in the regulation of MM progression.

Versican functions as a key modulator in tumor cell proliferation, migration and invasion. Increased expression of versican has been reported in multiple types of human malignancies, and has been associated with cancer relapse and poor survival rates in a number of cancer types, including breast and prostate (17). Furthermore, Touab *et al* showed that the expression of versican was intensely positive in primary and metastatic MM (18). Gambichler *et al* further reported that superficial spreading melanoma was associated with a significant overexpression of peritumoral versican (19). In the current study, the expression level of versican was also found to be markedly increased in MM tissues when compared with adjacent normal tissues, indicating that versican is involved in the pathogenesis of MM. In addition, silencing of versican promoted cell adhesion to type I collagen, laminin and fibronectin, indicating that versican plays proliferative, antiadhesive and promigratory roles in MM (12).

As the regulatory role of miRNA occurs predominantly via the expression inhibition of target genes, bioinformatic analysis was performed and versican was found to be a direct target of miR-203. Luciferase reporter assay results confirmed that miR-203 directly targeted the versican 3′-UTR at an evolutionarily conserved miR-203 binding site. The expression of versican has also been reported to be regulated by several miRNAs. For example, miR-138 and miR-199a were shown to directly target the 3′-UTR of versican mRNA, causing the inhibition of versican protein expression (20,21). However, the regulatory association between miRNA and versican is yet to be reported in MM. The present study further demonstrated that miR-203 negatively regulates the protein expression of versican in MM cells, but exhibits no effect on versican mRNA expression, indicating that miR-203 regulates versican expression at the post-transcriptional level. A number of targets of miR-203 have also been identified in MM. Noguchi *et al* showed that miR-203 induced senescence by targeting E2F3 in human MM cells (22). The authors also found that miR-203 reduced melanosome transport and promoted melanogenesis in MM cells by directly targeting KIF5B and inhibiting the cAMP response element-binding protein 1/microphthalmia-associated transcription factor/Rab27a pathway (9).

Furthermore, versican has been demonstrated to play a crucial role in the regulation of cancer cell migration (17). In versican-rich ECM, an antiadhesive effect is predominantly exerted, thus, cellular migration and the invasion of tumor cells is promoted (23,24). In addition, miR-203 has been reported to be downregulated in metastatic MM, while tumor cell migration is crucial for cancer metastasis (18). Accordingly, the present study focused on the effects of miR-203 and versican on MM cell migration. The observations revealed that miR-203 played an inhibitory role in the regulation of MM cell migration, while versican exhibited a promotional role. As miR-203 was found to negatively regulate the protein expression of versican in MM cells, whether the effect of miR-203 on MM cell migration was associated with versican was further investigated. The results indicated that upregulation of miR-203 significantly inhibited A375 cell migration, which was impaired by overexpression of versican, indicating that versican functions as a downstream effector in miR-203-mediated MM A375 cell migration.

In conclusion, the present study for the first time has identified versican as a novel target of miR-203 in MM cells. The results indicate that miR-203 plays an inhibitory role in MM cell invasion, partially at least, via the inhibition of versican. Therefore, versican may become a novel target for the inhibition of MM metastasis.

## Figures and Tables

**Figure 1:** miR-203 is downregulated in MM tissues and A375 cells. qPCR was performed to determine the expression levels of miR-203 in (A) 20 paired MM and matched adjacent tissue samples and (B) human MM A375 and normal skin HaCaT cells. T/N, tumor/normal; miR-203, microRNA-203, MM, malignant melanoma; qPCR, quantitative polymerase chain reaction.

**Figure 2:** Versican was identified as a novel target of miR-203. (A) Bioinformatic analysis demonstrated the putative seed region of miR-203 in the wild type 3′-UTR of versican. (B) A luciferase reporter assay was used to determine whether versican was a target of miR-203. Wild type and mutant type 3′-UTRs of versican were subcloned into a psiCHECK™2 reporter vector, which was cotransfected with 50 nM miR-203 or scramble negative control miRNA into A375 cells. ^**^P<0.01, vs. control. 3′-UTR, 3′-untranslated region; miR-203, microRNA-203.

**Figure 3:** Expression levels of versican were markedly upregulated in MM tissues. (A) qPCR was used to determine the mRNA expression of versican in 20 paired MM and matched adjacent normal tissue samples. (B) Western blot analysis was performed to determine the protein expression levels of versican in adjacent normal tissues and MM A375 cells; GAPDH was used as an endogenous reference. ^**^P<0.01, vs. normal. T/N, tumor/normal; MM, malignant melanoma; qPCR, quantitative polymerase chain reaction; GAPDH, glyceraldehyde-3-phosphate dehydrogenase.

**Figure 4:** miR-203 negatively regulated the expression of versican at a post-transcriptional level in A375 cells. (A) qPCR was used to determine the expression of miR-203 in A375 cells transfected with miR-203 mimics or miR-203 inhibitor; U6 was used as an endogenous control. ^**^P<0.01, vs. control. (B) Western blot analysis was used to determine the protein expression levels of versican in A375 cells transfected with miR-203 mimics or miR-203 inhibitor; GAPDH was used as an endogenous reference. ^*^P<0.05 and ^**^P<0.01, vs. control. qPCR, quantitative polymerase chain reaction; GAPDH, glyceraldehyde-3-phosphate dehydrogenase; miR-203, microRNA-203.

**Figure 5:** Effects of versican on MM A375 cell migration. (A) Western blot analysis was performed to determine the protein expression levels of versican in A375 cells transfected with versican plasmid or versican siRNA. (B) Cell migration analysis was performed using A375 cells transfected with versican plasmid or versican siRNA. ^**^P<0.01 vs. control. MM, malignant melanoma.

**Figure 6:** Versican functions as a downstream effector in miR-203-mediated MM A375 cell migration. A cell migration assay was performed using A375 cells transfected with miR-203 mimics, or cotransfected with miR-203 mimics and a versican plasmid. ^**^P<0.01. MM, malignant melanoma; miR-203, microRNA-203.

## References

[1] Trotter SC, Sroa N, Winkelmann RR, Olencki T, Bechtel M (2013). A global review of melanoma follow-up guidelines. J Clin Aesthet Dermatol.

[2] Linos E, Swetter SM, Cockburn MG, Colditz GA, Clarke CA (2009). Increasing burden of melanoma in the United States. J Invest Dermatol.

[3] Yates LA, Norbury CJ, Gilbert RJ (2013). The long and short of microRNA. Cell.

[4] Wagenseller AG, Shada A, D’Auria KM (2013). MicroRNAs induced in melanoma treated with combination targeted therapy of Temsirolimus and Bevacizumab. J Transl Med.

[5] Margue C, Philippidou D, Reinsbach SE (2013). New target genes of MITF-induced microRNA-211 contribute to melanoma cell invasion. PLoS One.

[6] Kozubek J, Ma Z, Fleming E (2013). In-depth characterization of microRNA transcriptome in melanoma. PLoS One.

[7] Yu X, Jiang X, Li H, Guo L, Jiang W, Lu SH (2014). miR-203 inhibits the proliferation and self-renewal of esophageal cancer stem-like cells by suppressing stem renewal factor Bmi-1. Stem Cells Dev.

[8] Wang C, Wang X, Liang H (2013). miR-203 inhibits cell proliferation and migration of lung cancer cells by targeting PKCα. PLoS One.

[9] Noguchi S, Kumazaki M, Yasui Y (2014). MicroRNA-203 regulates melanosome transport and tyrosinase expression in melanoma cells by targeting kinesin superfamily protein 5b. J Invest Dermatol.

[10] van Kempen LC, van den Hurk K, Lazar V (2012). Loss of microRNA-200a and c, and microRNA-203 expression at the invasive front of primary cutaneous melanoma is associated with increased thickness and disease progression. Virchows Arch.

[11] Wang X, Hu G, Zhou J (2010). Repression of versican expression by microRNA-143. J Biol Chem.

[12] Hernández D, Miquel-Serra L, Docampo MJ, Marco-Ramell A, Bassols A (2011). Role of versican V0/V1 and CD44 in the regulation of human melanoma cell behavior. Int J Mol Med.

[13] Choi E, Choi E, Hwang KC (2013). MicroRNAs as novel regulators of stem cell fate. World J Stem Cells.

[14] Hauptman N, Glavac D (2013). MicroRNAs and long non-coding RNAs: prospects in diagnostics and therapy of cancer. Radiol Oncol.

[15] Xu Y, Brenn T, Brown ER, Doherty V, Melton DW (2012). Differential expression of microRNAs during melanoma progression: miR-200c, miR-205 and miR-211 are downregulated in melanoma and act as tumour suppressors. Br J Cancer.

[16] Noguchi S, Mori T, Hoshino Y (2011). MicroRNAs as tumour suppressors in canine and human melanoma cells and as a prognostic factor in canine melanomas. Vet Comp Oncol.

[17] Du WW, Yang W, Yee AJ (2013). Roles of versican in cancer biology - tumorigenesis, progression and metastasis. Histol Histopathol.

[18] Touab M, Villena J, Barranco C, Arumí-Uría M, Bassols A (2002). Versican is differentially expressed in human melanoma and may play a role in tumor development. Am J Pathol.

[19] Gambichler T, Kreuter A, Grothe S (2008). Versican overexpression in cutaneous malignant melanoma. Eur J Med Res.

[20] Morton SU, Scherz PJ, Cordes KR (2008). microRNA-138 modulates cardiac patterning during embryonic development. Proc Natl Acad Sci USA.

[21] Lee DY, Shatseva T, Jeyapalan Z (2009). A 3′-untranslated region (3′UTR) induces organ adhesion by regulating miR-199a* functions. PLoS One.

[22] Noguchi S, Mori T, Otsuka Y (2012). Anti-oncogenic microRNA-203 induces senescence by targeting E2F3 protein in human melanoma cells. J Biol Chem.

[23] Du WW, Yang BB, Shatseva TA (2010). Versican G3 promotes mouse mammary tumor cell growth, migration, and metastasis by influencing EGF receptor signaling. PLoS One.

[24] Ween MP, Hummitzsch K, Rodgers RJ, Oehler MK, Ricciardelli C (2011). Versican induces a pro-metastatic ovarian cancer cell behavior which can be inhibited by small hyaluronan oligosaccharides. Clin Exp Metastasis.

